# Polyphenolic Fraction Obtained From *Thalassia testudinum* Marine Plant and Thalassiolin B Exert Cytotoxic Effects in Colorectal Cancer Cells and Arrest Tumor Progression in a Xenograft Mouse Model

**DOI:** 10.3389/fphar.2020.592985

**Published:** 2020-11-30

**Authors:** Livan Delgado-Roche, Kethia González, Fernando Mesta, Beatriz Couder, Zaira Tavarez, Ruby Zavala, Ivones Hernandez, Gabino Garrido, Idania Rodeiro, Wim Vanden Berghe

**Affiliations:** ^1^ Dirección Médica, Laboratorios Liomont S.A. de C.V., Ciudad de México, México; ^2^ Instituto de Ciencias del Mar (ICIMAR), La Habana, Cuba; ^3^ Escuela Nacional de Medicina y Homeopatía, Instituto Politécnico Nacional, Ciudad de México, México; ^4^ Universidad Nacional Autónoma de Mexico, Ciudad Universitaria, Ciudad de México, México; ^5^ Departamento de Ciencias Farmacéuticas, Facultad de Ciencias, Universidad de Católica del Norte, Antofagasta, Chile; ^6^ PPES Lab, Proteinchemistry, Proteomics and Epigenetic Signaling, Department of Biomedical Sciences, University of Antwerp, Antwerp, Belgium

**Keywords:** *T. testudinum*, polyphenols, thalassiolin B, colorectal cancer, reactive oxygen species, apoptosis

## Abstract

Marine plants are important sources of pharmacologically active metabolites. The aim of the present work was to evaluate the cytotoxic and antitumor activity of a polyphenolic fraction obtained from *Thalassia testudinum* marine plant and thalassiolin B in human colorectal cancer cells. Human cancer cell lines, including HCT15, HCT116, SW260, and HT29 were treated with tested products for cytotoxicity evaluation by crystal violet assay. The potential proapoptotic effect of these natural products was assessed by flow cytometry in HCT15 cells at 48 h using Annexin V-FITC/propidium iodide. In addition, reactive oxygen species (ROS) generation was measured by fluorescence using DCFH-DA staining, and sulfhydryl concentration by spectrophotometry. The *in vivo* antitumor activity of the polyphenolic fraction (25 mg/kg) was evaluated in a xenograft model in nu/nu mice. *In vivo* proapoptotic effect was also evaluated by immunohistochemistry using anti-caspase 3 and anti-Bcl-2 antibodies. The results showed that tested products exert colorectal cancer cell cytotoxicity. Besides, the tested products induced a significant increase (*p* < 0.05) of intracellular ROS generation, and a depletion of sulfhydryl concentration in HCT15 cells. The polyphenolic fraction arrested tumor growth and induced apoptosis in the xenograft mice model. These results demonstrate the cytotoxic activity of *T. testudinum* metabolites associated, at least, with ROS overproduction and pro-apoptotic effects. Here we demonstrated for the first time the antitumor activity of a *T. testudinum* polar extract in a xenograft mice model. These results suggest the potential use of *T. testudinum* marine plant metabolites as adjuvant treatment in cancer therapy.

## Introduction

Colorectal cancer (CRC) represents the fourth main cause of cancer death worldwide, with nearly 881,000 deaths in 2018 (Bray et al., 2018). The CRC progression implies a set of molecular events, including the activation of proto-oncogenes, inhibition of tumor suppressors, destruction of the cellular matrix, DNA mutations, and changes in DNA methylation state, most of them mediated by oxidative stress (OS) (Mayer, 2018). Inflammation caused by metabolic diseases, diet, and lifestyle factors, toxin, etc., increase the production of intestinal reactive oxygen species (ROS) (Pais and Dumitraşcu, 2018). ROS production is a key mechanism shared by most chemotherapeutics due to their implication in triggering cell death (Kim et al., 2012). Therefore, ROS induction has been considered a tumor-suppressing strategy widely described in the literature (Liou and Storz, 2010; Yang et al., 2018). Under physiological conditions, a certain ROS level contributes to maintain the delicate balance between proliferation and apoptosis of cells. In these conditions, low ROS levels can activate tyrosine kinases and NF-κB signaling pathways and hypoxia-inducible factor, which participate in cell growth processes. On the contrary, excessive ROS levels may activate signaling cascades which inhibit cell growth and proliferation, and induce apoptosis (Qiu et al., 2020). In addition, the intracellular increase of ROS levels in cancer cells promotes genome instability, which can induce cell cycle arrest and inhibition of cell proliferation. Therefore, ROS-based therapies have been proposed and widely evaluated as a chemopreventive strategy to arrest tumor progression (Wang et al., 2017a).

The above-mentioned line of evidence has increasingly led to studies aimed toward the identification of novel compounds, preferably from natural sources having anti-cancer potential with minimal collateral damages to normal cells. Polyphenols are known to elicit cancer selective cytotoxic effects (Pampaloni et al., 2014; Jiménez et al., 2016; Zhou et al., 2018), in more particular apoptosis cell death (Brusselmans et al., 2005; Kim et al., 2006; Yi et al., 2016).

*Thalassia testudinum* seagrass (*T. testudinum*) has potential therapeutic use (Garateix et al., 2011; Regalado et al., 2012; García et al., 2017; Riera et al., 2018; Rodeiro et al., 2018), which in a near future can be approached as a nutraceutical product. The phytochemical characterization of an aqueous-ethanolic extract as well as the polyphenolic fraction from *T. testudinum* grown in the Cuban coasts showed a complex mixture containing phenols, flavonoids, proanthocyanidins, among others structures with cytotoxic effects (Table 1) (Regalado et al., 2012; Rodeiro et al., 2018; Riera et al., 2018). The glycosylated sulphated flavone thalassiolin B (chrysoeriol 7-β-D-glucopyranosyl-2"-sulphate) (TB) has been identified as the main component found in *T. testudinum* hydroethanolic extract (5.8% w/w) (Figure 1) (Regalado et al., 2009; Garateix et al., 2011; Regalado et al., 2012). Recent work of our group provided evidence of the cytotoxic and DNA damage of the crude extract of *T. testudinum* on tumor cell lines. Additionally, this work suggested that the cytotoxic effect of the extract is associated with OS, nuclear damage, and sustained hypercalcaemia in HepG2 cells (Rodeiro et al., 2018). Along the same line, a chloroform fraction from *T. testudinum* was found to elicit cytotoxicity and antiproliferative effects on A549 and EA.hy926 immortalized cells as well (Riera et al., 2018). Altogether, these results demonstrate promising antitumor properties of the polyphenolic fraction of *T. testudinum* (PF) and TB, which could be confirmed in a xenograft mice model, a relevant animal model of human cancer research.

**TABLE 1:** Chemical components in *T. testudinum* polyphenolic extract.

Components	% ± SD^a^	Compounds identified
Total polyphenols	29.5 ± 1.2	ethyl 4-(sulfooxy)benzoate, 4-hydroxybenzoic acid, 4-hydroxybenzaldehyde, chrysoeriol-7-O-D-glucopyranosyl-2-sulfate (thalassiolin B), apigenin 7-O-D-glucopyranosyl-2-sulfate (thalassiolin C), chrysoeriol 7-O-Dglucopyranoside, apigenin 7-O-D-glucopyranoside, 5,7-dihydroxy-3',4'-dimethoxyflavone 7-O-D-glucopyranoside, luteolin-3'-sulfate, chrysoeriol, apigenin
Proanthocyanidins	21.0 ± 2.3	—
Flavonoids	4.6 ± 0.2	—
Polysaccharides	5.8 ± 1.6	—
Soluble proteins	16.2 ± 0.7	—

a Values are expressed as g per 100 g of the dry extract (%, w/w). Thalassiolin B represents 5.8 ± 0.3 of total extract (Regalado et al., 2012; Rodeiro et al., 2018).

**FIGURE 1:** Chromatographic profile of thalassiolin B isolated from *T. testudinum* hydroethanolic extract. **(A)** Chemical structure of thalassiolin B (chrysoeriol 7-β-D-glucopyranosyl-2"-sulphate), the main component of *T. testudinum* extract. **(B)** HPLC of thalassiolin B standard. **(C)** HPLC profile of *T. testudinum* hydroethanolic extract. Adapted from: Garateix et al., 2011. The authors have the rights to share this figure.

## Materials and Methods

### Plant Material

*T. testudinum* (Banks and Soland ex. Koenig) was collected during March 2016 in “Guanabo” beach (22° 05’ 45’’ N, 82° 27’ 15’’ W), previous authorization to access plant samples by Cuban Office for Environmental Regulatory. The specimen was identified by Dr. J. A. Areces (Institute of Oceanology, Havana, Cuba) and a voucher sample (IDO No.39) was deposited in the herbarium of the Cuban National Aquarium. Whole dry and ground *T. testudinum* leaves (840 g) were continuously extracted with EtOH-H_2_O (50:50, v/v) during 24 h at room temperature. The extract was filtered and concentrated under reduced pressure and temperature (40°C) to yield 54 g of crude extract. The crude extract was used to obtain a polyphenol-rich fraction, where non-polar components were excluded by chloroform extraction (1:10, w/v). The polar fraction was filtered and dried at room temperature. TB (1-chrysoeriol 7-β-D-glucopyranosyl-2″-sulphate) was isolated also from the extract by electrospray ionization mass spectrometry (ESIMS) with an [M-H]—ion at m/z = 541. Its structure was confirmed by spectroscopic analysis (^1^H and ^13^C nuclear magnetic resonance (NMR), gCOSY60, gHSQC, gHMBC, ROESY experiments) and compared to reported data (Rowley et al., 2002).

### Cell Lines

The human colon carcinoma cells HCT15 (RRID:CVCL-0292), HCT116 (RRID:CVCL-0291), HT29 (RRID:CVCL-0320), SW620 (RRID:CVCL-0547), and human normal cells FHC (RRID:CVCL-3688), HEL299 (RRID:CVCL-2480), MCF10A (RRID:CVCL-0598) were obtained from American Type Culture Collection (ATCC, Manassas, United States) and maintained in proper culture media as indicated.

### Cell Viability by Violet Crystal Assay and Selective Index

Cancer cells HCT15, HCT116, HT29, SW620 and normal cells FHC, HEL299 and MCF10A were seeded in 48-well plates at a density of 4 × 10^4^ viable cells/cm^2^ in DMEM + 10% FBS. Cells were incubated for 24 h in 5% CO_2_ atmosphere and 95% humidity at 37°C. Then, the cells were treated with PF and TB (2.5–500 µg/ml), camptothecin (0.25–10 µM) for 24 and 48 h. As control, (100 cell viability), cells were maintained in culture media. After treatments, cells were washed with sterile PBS and fixed with DMEM/F12, SFB 2%, and glutaraldehyde 1.1% for 15 min at room temperature. Afterward, the fixation medium was removed, the cells were dried, and 200 µl of crystal violet solution (0.5%) was added during 15 min at room temperature. Finally, the crystal violet was removed, and the stained cells were resuspended in 500 µl of 10% acetic acid (Feoktistova et al., 2016). The absorbance was recorded at 595 nm in a microplate reader (Bio-Rad, Mexico). The tests were carried out in two independent experiments by triplicate. Results were expressed as percentage cell viability respect to non-treated cells (assumed as 100% value), using the following equation: Cell viability (%) = 100–[(Absorbance control–Absorbance test/Absorbance control) × 100]. IC_50_ (concentration of the compounds that is required for 50% inhibition cell viability) values were determined from the best-fit of the Hill slope curve to experimental data using nonlinear regression analysis by using five different sample concentrations. To determine the cytotoxic selectivity index of products, the selectivity index (SI) was determined using the formula: SI = IC_50_ of non cancer cell/IC_50_ of cancer cell, where a SI ≥ 10 was considered a selective compound (Peña-Morán et al., 2016).

### Flow Cytometry

Cell apoptosis was measured in the most sensitive cells HCT15 by annexin V-fluorescein isothiocyanate (FITC)/propidium iodide staining (GTX85591, GeneTex, United States). Briefly, HCT-15 cells were incubated with PF or TB (mean IC_50_ = 22.47 µg/ml and 38.75 µg/ml, respectively), cisplatin (10 µM) or media for 48 h. Treated cells were collected by trypsinization and centrifuged at 1,500 rpm during 5 min, washed with cold PBS, and resuspended in diluted binding buffer. Afterward, cells were stained with a mixture of FITC-annexin-V (5 µl) and propidium iodide solution (5 µl) in binding buffer (500 µl) and incubated for 5 min at room temperature in the dark condition. Then, cells were centrifuged, re-suspended in 1 ml assay binding buffer, and analyzed by Fluorescence Activated Cell Sorting (BD FACS Aria II, BD Biosciences, United States) within 1 h following the staining. A minimum of 10,000 cells was analyzed per experimental group. The data acquisition and analysis were performed using BD CellQuest Pro Software.

### Measurement of Reactive Oxygen Species Generation

The intracellular ROS level was assessed in HCT15 cell cultures by 2′,7′-dichlorofluorescin diacetate (DCFH-DA) staining. In brief, cells were incubated with PF (22.47 µg/ml), TB (38.75 µg/ml), or cisplatin (10 µM) for 24 h. N-acetylcysteine was added to the cell media 1 h before PF and TB. Then, cells were washed with phosphate buffer saline (PBS, pH = 7.4) and incubated with DCFH-DA (20 mM) for 20 min in the dark at 37°C. Fluorescence was recorded using a BD Bioscience Fluorescent Microscope, (US) at an excitation wavelength of 490 nm and an emission wavelength of 525 nm.

### Measurement of Sulfhydryl Concentration

The intracellular sulfhydryl (−SH) concentration was determined in HCT15 cells using a commercial kit (Cayman Chemical Co., Ann Arbor, MI) after 24 h treatment with test compounds in a visible UV plate reader (Pharmacia, United States) at 405 nm.

### Toxicological Assessment in Mice

Nu/Nu female mice (*n* = 3) fasted for 10 h prior to dosing were exposed to intraperitoneal (i.p) doses of *T. testudinum* extract and TB (25 and 250 mg/kg). Test doses were selected according to the pharmacological studies, covering an adequate safety margin. As negative control three mice received PBS i.p., meanwhile the positive control group (*n* = 3) received cisplatin 2 mg/kg (i.p.). The test products were administered three times a week for 21 days. The body weight and behavior of mice were monitored every third day during treatment. Mice were euthanized on day 21 by intraperitoneal administration of pentobarbital (50 mg/kg). Histological examination (hematoxylin-eosin staining) were performed in the Department of Pathology, Faculty of Veterinary Medicine (UNAM, Mexico City, Mexico) under standard procedures.

### Antitumor Effect of *T. testudinum* Polyphenolic Fraction in Mice

Male Balb/c nu/nu nude mice (CAnN.Cg-*Foxn1*^*nu*^/Crl Immunodeficient Inbred), 6–8 weeks old, weighing 18–24 g, were used to establish the HCT-15 xenograft tumor model. The animals (n = 15) were purchased from Charles River Laboratories (San Francisco, CA, United States) and keep in quarantine for 15 days. The mice were housed in laboratory animal barrier systems under specific pathogen-free conditions with controlled temperature and humidity, and exposed to 12 h light/dark cycle (five animals per cage). The experimental protocol (ID249) was previously approved by the Institutional Ethical Committee of the Instituto de Investigaciones Biomédicas (Mexico City, Mexico). The xenograft model of HCT15 was established by a subcutaneous (s.c.) injection of 2 × 10^6^ HCT15 cells/100 µl into the lower right flank region. On day 3, when tumors were sized between 30 and 50 mm^3^, mice were randomly distributed in three groups (*n* = 5). The first group (control group) was orally treated with PBS three days a week for 27 days, the second group was orally treated with PF (25 mg/kg) three days a week for 27 days, and the third group (control group) was intraperitoneally treated with cisplatin (2 mg/kg) 3 days a week for 27 days. Tumor size was evaluated by two measurements, a = length and b = width, with a calibrated slide caliper. Values of tumor volume (mm^3^) were determined as previously described [24], V= (a × b^2^)/2 (Kersemans et al., 2013). At the end of the experiment, serum samples were obtained for biochemical determinations. Finally, mice were euthanized by the intraperitoneal administration of pentobarbital (50 mg/kg).

### Immunohistochemistry Analysis

Representative tumor sections were fixed in a 10% formaldehyde solution for 24 h and embedded in paraffin. Four-micrometer tissue sections were deparaffinized, rehydrated, and blocked for endogenous peroxidase activity; then, tissue sections were immunostained with primary antibody for caspase 3 and Bcl2 proteins (Abcam) overnight at 4°C. Finally, staining with the DAB detection kit (Sigma Aldrich, United States) and counterstained with hematoxylin (Sigma-Aldrich). Immunostained sections were captured in an Olympus BX51 optical light microscope were quantified using computerized image analysis (Adobe Photoshop CS4 software).

### Serum Oxidative Stress Biomarkers

Malondialdehyde (MDA) content was determined in serum samples, as previously described (Erdelmeier et al., 1998). Protein carbonyl groups were determined by using a commercial kit (Cayman, MI, United States) based on the 2,4-dinitrophenylhydrazone (DNPH) method (Levine et al., 1994). Superoxide dismutase (SOD) activity was determined by using a commercial kit (Randox Labs, United Kingdom), where xanthine and xanthine oxidase were used to generate superoxide anion radicals (O_2_^•−^), which react with 2-(4-iodophenyl)-3-(4-nitrophenol)-5-9 phenyltetrazolium chloride to form a red formazan dye. Catalase (CAT) activity was determined by following the decomposition of hydrogen peroxide (H_2_O_2_) at 240 nm (Aebi, 1984).

### Statistical Analysis

Data are represented as mean ± standard deviation (SD). Statistical differences were determined using SPSS version 24.0 (IBM, United States). Multiple comparisons were carried out by one-way ANOVA followed by a Tukey *post-hoc* test. All comparisons are made concerning untreated controls. Statistical significance was set as *p < 0.05.

## Results

### Polyphenolic Fraction and Thalassiolin B Exert Cytotoxicity Activity

Crystal violet assay showed a reduction of survival percentage of cancer cells exposed to test products in a time and dose-dependent manner (data not shown). The most sensitive cell line to treatments was HCT15, showing IC_50_ values at 48 h in the order of 22.47 ± 1.30 µg/ml and 38.75 ± 3.57 µg/ml for PF and TB, respectively. The selectivity index (>10) suggest a high selectivity of the tested compounds in this cell line (Table 2). Of note, the products did not show cytotoxic effects on normal human cells (data not shown).

**TABLE 2:** Cytotoxicity and selectivity evaluation of *T. testudinum* extract and thalassiolin B in different human colorectal cancer cell lines.

Test products	Colorectal cancer cell lines			
	HCT15	HT29	SW620	HCT116
	Treatment 24 h			
PF IC_50_ (µg/ml) *(SI)*	36.51 ± 4.68 *(17.80)*	101.46 ± 9.22 *(6.40)*	>500 *(1.12)*	>500 *(1.04)*
TB IC_50_ (µg/ml) *(SI)*	51.82 ± 8.72 *(12.54)*	136.61 ± 10.28 *(4.76)*	>500 *(0.96)*	>500 *(0.75)*
Camptothecin IC_50_ (µM) *(SI)*	8.11 ± 0.92 *(1.11)*	6.71 ± 2.01 *(1.25)*	8.09 ± 2.31 *(1.11)*	6.23 ± 2.56 *(1.44)*
**Treatment 48 h**				
PF IC_50_ (µg/ml) *(SI)*	22.47 ± 1.30 *(28.92)*	93.11 ± 4.05 *(6.98)*	>500 *(1.04)*	>500 *(1.02)*
TB IC_50_ (µg/ml) *(SI)*	38.75 ± 3.57 *(16.75)*	121.71 ± 3.41 *(5.34)*	>500 *(0.90)*	>500 *(0.80)*
Camptothecin IC_50_ (µM) *(SI)*	6.82 ± 0.88 *(1.61)*	7.21 ± 1.19 *(1.51)*	7.88 ± 1.92 *(1.40)*	6.77 ± 2.13 *(1.62)*

Values represent mean ± standard deviation values of IC_50_ (concentration of tested products that inhibits the 50% of cell viability after 24 and 48 h exposure). Cell viability was assessed by crystal violet assay using camptothecin (0.25–10 µM) as reference cytostatic compound and test product (2.5–500 µg/ml). Three independent experiments by quadruplicate were carried out. SI: selectivity index was calculated as the ratio of IC_50_ in normal cells (FHC cells)/IC_50_ in cancer cells. SI ≥ 10 was considered a selective compound.

### Polyphenolic Fraction and Thalassiolin B Induce HCT15 Cells Apoptosis

Untreated and treated HCT15 cells were stained with annexin-V/FITC and propidium iodide (PI) and analyzed by flow cytometry for detecting phosphatidylserine externalization during the apoptosis process. Representative histograms of flow cytometry assays are shown in Figures 2A. A significant increase in the number of apoptotic cells was observed at IC_50_ values of tested products. The mean percentage of cells in the early and late apoptosis population at 48 h was 9.97 and 34.08% for PF; meanwhile, for TB the mean percentage of apoptotic cells was 10.75 and 44.51%, respectively (Figures 2A,B). Of note, the increment of late apoptotic cells population was significantly higher (*p* < 0.05) in PF and TB treated cells compared with cisplatin treated cells (early apoptosis: 50.33%; late apoptosis: 15.99%) (Figures 2A,B). The mean percentages of necrotic cells were not significant in any of the treated groups.

**FIGURE 2:** Apoptosis of HCT15 cells after 48 h of exposure to the polyphenolic fraction and thalassiolin B obtained from *T. testudinum* extract (at IC_50_ values). **(A)** Representative histogram of flow cytometry analysis by annexin V-FITC/propidium iodide staining. **(B)** Analysis of the percentage of apoptotic cells in each group. Cisplatin (10 µM) was used as positive control. PF, polyphenolic fraction; TB, thalassiolin **(B)**. Bars represent the mean ± standard deviation of two independent experiments by triplicate. Different symbols represent statistical differences between groups (one-way ANOVA, followed by Tukey *post-hoc* test, *p* < 0.05).

### Polyphenolic Fraction and Thalassiolin B Induce Reactive Oxygen Species Generation and Antioxidant Depletion in HCT15 Cells

The potential effect of tested products on intracellular ROS generation was evaluated by DCFH-DA staining. PF and TB, at IC_50_ values, induced a significant increase (*p* < 0.05) of intracellular ROS (Figures 3C,D) as suggested by the high fluorescence units at 24 h. When cells were pre-treated with N-acetylcysteine prior to the test products, the fluorescence was significantly reduced (*p* < 0.05) compared with cells only treated with PF or TB (Figures 3E,F). Together with the increment of intracellular ROS in PF and TB treated cells, a significant reduction (*p* < 0.05) of total sulfhydryls was observed in comparison to untreated HCT15 cells (Figures 3H).

**FIGURE 3:** Intracellular reactive oxygen species generation and sulfhydryl levels in HCT15 cells after 24 h of exposure to the polyphenolic fraction and thalassiolin B from *T. testudinum* extract (at IC_50_ values). **(A)** control cells; **(B)**: cisplatin (10 µM); **(C)**: polyphenolic fraction; **(D)**: thalassiolin B; **(E)**: N-acetylcysteine + polyphenolic fraction; **(F)**: N-acetylcysteine + thalassiolin **(B)**. Bars represent mean ± standard deviation of fluorescence arbitrary units **(G,H)**. Two independent experiments by triplicate were carried out. Different symbols on bars represent statistical differences (ANOVA, Tukey *post-hoc*, *p* < 0.05).

### Polyphenolic Fraction and Thalassiolin B are Safe and Well Tolerated by nu/nu Female Mice

No signs of toxicity were observed during the toxicological evaluation. A normal tendency in body weight gains were observed in animals of control group and in those where PF and TB were administered. In contrast, the body weight was significantly reduced at the end of the experiment in cisplatin treated animals (*p* < 0.05), considered as a clear sign of drug toxicity (Figures 4B). Macroscopic and microscopic examination of organs and tissues did not reveal abnormal findings in treated animals, except for cisplatin group (Figures 4A). These results suggest that natural extracts (at tested doses) are less toxic than cisplatin and well tolerated by nu/nu female mice.

**FIGURE 4:** Toxicity assay of PF and TB in nu/nu female mice. **(A)**: representative slides of H&E statining of different organs including liver, spleen and kidney. **(B)**: time-course of body weight in different groups. Group 1: control (PBS, i.p.); group 2: cisplatin (2 mg/kg, i.p.); group 3: PF (25 mg/kg, i.p.); group 4: PF (250 mg/kg, i.p.); group 5: TB (25 mg/kg, i.p.); group 6: TB (250 mg/kg, i.p.). Bars: 50 µm, magnification ×20.

### Polyphenolic Fraction Arrest Tumor Growth

To explore the potential antitumor effect of PF, we developed an HCT15 xenograft model in nude mice. When tumor volume was higher than 30 mm^3^, the animals were orally treated with PF (25 mg/kg) or intraperitoneal dose of cisplatin (2 mg/kg) 3 days a week for 27 days. All the animals were included in the analysis. The repeated dose of cisplatin significantly (*p* < 0.05) diminished the animal body weight; meanwhile, PF did not affect the treated animals (Figures 5D). Our results showed an arresting tumor progression by PF treatment, as demonstrated in the significant reduction (*p* < 0.05) of tumor volume and weight (Figures 5B–F). At the end of the experiment, the group receiving PF showed a high survival rate compared with control and cisplatin groups (Figures 5C). In addition, lipid peroxidation, measured by MDA levels, were significantly lower (*p* < 0.05) when compared with control and cisplatin-treated mice. Total protein carbonyl groups, were significantly diminished (*p* < 0.05) respect to the animals intraperitoneally treated with cisplatin; meanwhile, no differences (*p* > 0.05) were observed when compared with the control group. The antioxidant enzyme activities were significantly lower (*p* < 0.05) in cisplatin, and PF treated animals respect to control animals; however, the enzymatic activity of SOD and CAT was higher (*p* < 0.05) in PF receiving mice respect to those treated with cisplatin (Table 3). Also, the immunohistochemical analysis revealed a significant increment (*p* < 0.05) of caspase 3 and Bcl-2 protein expression in the animal treated with PF and cisplatin compared with control mice (Figure 6).

**FIGURE 5:** Antitumor effect of the polyphenolic fraction from *T. testudinum* extract in nu/nu mice. Animals (*n* = 5) were orally treated for 27 days with the polyphenolic fraction (25 mg/kg), or intraperitoneally with cisplatin (4 mg/kg) after xenograft model of HCT15 was established **(A)**. Control group: animals treated with oral doses of PBS. Representative tumoral mass after mice’s euthanasia **(B)**. Mean ± standard deviation of tumor volume and weight **(E**,**F)**. Survival rate and body weight **(G)** behavior during the experiment **(C**,**D)**.

**TABLE 3:** Effects of *T. testudinum* extract on systemic oxidative stress in nu/nu mice.

Biomarkers	Control group (*n* = 5)	Cisplatin (2 mg/kg) (*n* = 5)	PF (25 mg/kg) (*n* = 5)
MDA (µmol/L)	9.27 ± 1.02	11.67 ± 2.11^a^	6.34 ± 0.97^a^
Carbonyls (µmol/l)	2.03 ± 0.52	6.73 ± 0.88^a^	2.92 ± 1.01
SOD (U/ml)	68.00 ± 14.21	22.00 ± 9.34^a^	49.00 ± 7.66^a^
CAT (U/ml)	1,125.00 ± 42.74	723.00 ± 51.20^a^	911.14 ± 31.26^a^

Values represent mean ± standard deviation values of serum biomarkers of oxidative stress. MDA, malondialdehyde; SOD, superoxide dismutase; CAT, catalase. Serum samples were analyzed by triplicate on two different days.

a Statistical differences respect control animals (ANOVA, Tukey *post-hoc*, *p* < 0.05).

**FIGURE 6:** Caspase 3 and Bcl-2 expression in tumoral tissue of nu/nu mice. Representative slides of cleaved caspase 3 expression and Bcl-2 in tumoral tissue determined by immunohistochemistry technique (five animals per group). Bar graphs represent the densitometry analysis of cleaved caspase 3 positive area/total area (%) and Bcl-2 positive area/total area (%). Bars: 50 µm, magnification ×20. Bars in the graphs represent the mean ± standard deviation of percentages. Asterisks represent statistical differences between groups (one-way ANOVA, followed by Tukey *post-hoc* test, *p* < 0.05).

## Discussion

The growing need to develop new antitumoral drugs with lesser unspecific cytotoxicity and side effects has fueled exploration of new sources of pharmacologically active compounds from natural products with a broad range of antitumor mechanisms (Bishayee and Sethi, 2016; Cragg and Pezzuto, 2016). The polypharmacological approach to the treatment of complex diseases has been a concept that has gained increased attention in recent years (Ho et al., 2018; Saqib et al., 2018). In this line, dietary polyphenols are naturally occurring compounds with different biological activities and mechanisms such as antioxidant (Zhang and Tsao, 2016), anti-inflammatory (Yahfoufi et al., 2018; Khan et al., 2020), and anti-carcinogenic properties (Nikš and Otto, 1990). Thus, dietary polyphenols may represent attractive nutraceutical alternatives, especially as co-treatment or adjuvant of anticancer drugs. Accordingly, in the present work, we evaluated the antitumor effect of polyphenolic components from *T. testudinum* and a pure constituent phytochemical TB, as well as their potential underlying molecular mechanisms.

Here, we observed a selective cytotoxic effect of PF and TB on cancer cell lines, in particular HCT15 cells, since more than 95% of viability was observed in normal human cell lines (FHC, HEL299 and MCF10A) up to 500 µg/ml (data not shown). *In vitro* studies have extensively demonstrated antitumor activity of polyphenols in different cancer cell lines by means of cell viability/toxicity assays, e.g., MTT assay (Vichai and Kirtikara, 2006), Sulforhodamine B assay (Mericli et al., 2017) and Crystal Violet method (Feoktistova et al., 2016). Cytotoxic effects of *T. testudinum* aqueous-ethanolic extract were previously demonstrated in HepG2, PC12, Caco-2 and 4T1 cell lines. In the hepatoma cells, the cytotoxic effect was partially associated with OS, nuclear DNA damage and hypercalcemia mechanisms (Rodeiro et al., 2018). Recently, non-polar components of *T. testudinum* extract were characterized and evaluated as potential cytotoxic compounds. By GC-MS methods, approximately 69 compounds of the non-polar fraction were identified, where fatty acids, mainly palmitic acid, were the major components. The cytotoxic potential of this chloroform fraction was observed in A549 and EA.hy926 (Riera et al., 2018). Many reports have demonstrated the cytotoxic activity of fatty acids from vegetal sources in tumoral cell lines, including colorectal cancer cells (Mileo and Miccadei, 2016; Yang et al., 2017; Pacheco et al., 2018; Devanadera et al., 2019).

To date, the cytotoxic and potential antitumoral mechanisms of PF and TB are not fully understood. However, one of the most accepted mechanisms underlying the cytotoxicity of polyphenols is the ROS-induced cancer cell apoptosis (Wang et al., 2017a, Wang et al., 2017b). Here we showed that PF and TB induced an increase of intracellular ROS in HCT15 cells, together with deprivation of sulfhydryl levels, suggesting increased levels of OS (Figure 3). Compared to the normal cells, cancer cells are more prone to collapse by ROS attack, since malignant cells already show elevated levels of OS in unexposed conditions, which limits their buffering capacity (Wang et al., 2017a, Wang et al., 2017b). As previously reported, *T. testudinum* extract increases the cytosolic Ca^2+^ concentration, triggering ROS generation and DNA fragmentation. These effects were associated with reduced cell viability (Rodeiro et al., 2018). High levels of ROS damage nuclear DNA and mitochondria, leading to the activation of apoptosis (Derdak et al., 2008; Wang et al., 2017a, Wang et al., 2017b). High levels of antioxidants and ROS suppressors have been found to promote chemoresistance in tumoral cells (Hernández et al., 2015). Hence the induction of further OS by dietary polyphenols in cancer cells holds promise to sensitize tumors to chemotherapy.

Besides the increased generation of intracellular ROS in HCT15 cells, we demonstrated that tested products induce apoptosis cell death. The externalization of phosphatidylserine was confirmed by flow cytometry analysis. Despite limitations to further explore the impact of tested products on other mediators of cell apoptosis, these results represent the first evidence suggesting the potential pro-apoptotic effect of polyphenolic components of *T. testudinum* extract and its main component, TB in cancer cells. However, it is well stablished that high levels of ROS can activate mitochondrial, death receptor and endoplasmic reticulum pathways of apoptosis. Here, we observed that *T. testudinum* and TB induced the generation of high levels of intracellular ROS in HCT15 cells. Therefore, these results preliminarily suggest a possible intrinsic apoptosis pathway activation, since Bcl-2 expression was increased in the tumoral tissue of animals treated with PF or cisplatin (Redza-Dutoirdoir and Averill-Bates, 2016). This hypothesis should be further demonstrated in future studies.

We further examined the *in vivo* antitumor effect of PF in an HCT15 xenograft mice model. Mice were treated with 25 mg/kg of PF during 27 days, based on previous dose response experiments (Hernández et al., 2015). Following PF treatment, we observed a significant reduction of tumor volumes and weights as compared to control mice. Meanwhile, no significant differences of animal survival were observed between groups at the end of the experiment. In contrast to cytotoxic levels of OS in tumor cells, systemic OS biomarkers were decreased in PF-treated animals, which may be associated with antioxidant scavenging properties of phytochemicals present in the *T. testudinum* extract. Epidemiological studies suggest that dietary polyphenols could reduce systemic OS levels and inflammation, attenuating the CRC risk. In addition, the potential role of natural polyphenols in increasing the cell sensitivity to colon cancer chemotherapy has been linked with a relevant improvement of cancer treatment (Wang et al., 2013; Schwingshackl et al., 2017; Mileo et al., 2019).

In summary, these results altogether demonstrate the cytotoxic activity of a polyphenolic rich fraction and TB obtained from the marine angiosperm plant *T. testudinum* in human CRC cell lines. In addition, the *in vivo* antitumor effect of this natural product is reported for the first time in a xenograft mouse model. Moreover, we identified the critical involvement of OS and apoptosis in the antitumor activity of *T. testudinum* metabolites. Altogether, these results favor the potential use of *T. testudinum* marine plant as a novel nutraceutical adjuvant in colon cancer therapy.

## Data Availability Statement

The raw data supporting the conclusions of this article will be made available by the authors, without undue reservation.

## Ethics Statement

The animal study was reviewed and approved by Institutional Animal Care and Use Committee of the Instituto de Investigaciones Biomédicas, Universidad Nacional Autónoma de México, Mexico City, Mexico.

## Author Contributions

IR and LD-R were responsible for the general study concept, conducting experimental analysis, interpreting and discussing of results, and drafting the manuscript. LD-R, KG, FM, BC, and ZT contributed, analyzed and interpreted the chemical and biological experiments. WB and GG contributed to the study concept and discussing of results. FM carried out statistical data analysis. IH and RZ were the study coordinators. Funding acquisition: IR, GG, and WB. All authors have read and approved the final manuscript.

## Funding

This work was supported by the research projects: CITMA P211LH005-051 (Cuba), the Project FONDECYT 1130601 (Chile) and the VLIR TEAM/Own Initiatives-Programme 2016 ZEIN2016PR420 project (Belgium). Dr. Delgado-Roche received a posdoc scholarship from “*Becas de Excelencia del Gobierno de México para Extranjeros 2016*” (AMEXCID, Mexico).

## Conflict of Interest

The authors declare that the research was conducted in the absence of any commercial or financial relationships that could be construed as a potential conflict of interest.
